The article "Continuous Renal Replacement Therapy for Hypertension Complicated by Refractory Heart Failure: An Analysis of Safety and Nursing Highlights" was retracted in 2023. Reasons: signs of a paper mill; compromised peer review; unreliable results or conclusions.

# Continuous Renal Replacement Therapy for Hypertension Complicated by Refractory Heart Failure: An Analysis of Safety and Nursing Highlights

**DOI:** 10.1155/2022/7951744

**Published:** 2022-09-14

**Authors:** Miaoli Zhang, Jingfeng Li

**Affiliations:** Department of Fourth Cardiovascular Medicine, The Affiliated Chuzhou Hospital of Anhui Medical University, The First People's Hospital of Chuzhou, Chuzhou, Anhui 239000, China

## Abstract

**Objective:**

This research is aimed at analyzing the safety profile and nursing highlights of continuous renal replacement therapy (CRRT) for hypertension (HT) complicated by refractory heart failure (RHF).

**Methods:**

Sixty-six HT + RHF patients admitted between March 2018 and December 2021 were enrolled and assigned to two groups: a CRRT group with 33 cases treated with CRRT and a control group with 33 cases intervened by routine treatment. The therapeutic effect and alterations of cardiac function (CF) indexes were observed in both cohorts. Besides, statistics were made in terms of serum B-type natriuretic peptide (BNP), C-reactive protein (CRP) and mean arterial pressure (MAP) concentrations, time of asthma relief, heart rate recovery (HRR), edema resolution, and hospitalization, as well as incidence of adverse reactions (ARs). Finally, pre- and posttreatment psychological quality and pain of both cohorts of subjects were assessed using the self-rating anxiety and depression scale (SAS and SDS) and visual analogue scale (VAS), respectively.

**Results:**

CRRT group exhibited higher overall response rate and better CF than control group (*P* < 0.05), with lower BNP, CRP, and MAP levels, and shorter time of asthma relief, HRR, edema resolution, and hospitalization (*P* < 0.05); the incidence of ARs was similar (*P* > 0.05); for both groups, the scores of SAS, SDS, and VAS reduced statistically after treatment (*P* < 0.05).

**Conclusion:**

CRRT can effectively improve the therapeutic effect and CF of patients with HT complicated by RHF, to protect the health and safety of patients.

## 1. Introduction

Hypertension (HT) is an extremely prevalent chronic disease among the middle-aged and elderly; the clinical manifestations are paroxysmal or persistent dizziness, headache, insomnia, memory loss, and limb numbness, which have a serious impact on the quality of life and physical and mental health of patients [1]. Cardiocerebral disorders and renal dysfunction are common complications in hypertensive patients [2]. HT has been confirmed as the major risk factor for heart failure (HF), and due to the high age of hypertensive patients and the deterioration of physical functions, HF often develops into refractory critical diseases, and it is manifested as continuous aggravating palpitations, dyspnea, chest tightness, asthma, etc., which eventually lead to large-area myocardial infarction or myocardial fibrosis, posing a serious threat to patients' life safety [3]. Refractory heart failure (RHF) is in the severe stage of HF, when the renal blood flow is significantly reduced, accompanied by abnormal blood flow distribution, renal interstitial edema, and obviously decreased glomerular filtration rate, which can directly cause acute renal failure in severe cases [4]. This process can also lead to a substantial decline in cardiac output, most of which are accompanied by compensatory enhancement of neurohumoral factor activity and vasoconstriction, further increasing the cardiac load and aggravating the pathological development of RHF [5]. Therefore, correcting the renal blood flow in RHF is of great significance for disease treatment. Affected by RHF, the sensitivity of the patient's kidney to diuretics is greatly reduced that has been unable to meet the treatment requirements [6]. Besides, due to the influence of neuroendocrine system activation, diuretic resistance, electrolyte disorder, and other factors, there is an urgent need to find a safer and more effective treatment in clinical practice [7].

At present, comprehensive treatment is mostly adopted for the clinical treatment of HT complicated by RHF clinically (HT + RHF); although it has certain therapeutic effect, the occurrence of adverse reactions (ARs) in the long-term treatment process worsens the final prognosis of patients [8, 9]. Therefore, the clinic is urgently looking for a more effective RHF treatment method, to protect the life safety of patients. With the continuous progress of medical technology, continuous renal replacement therapy (CRRT) has gradually become an important therapy for the treatment of critical diseases. Through extracorporeal circulation blood purification technology, water and solute are continuously and slowly removed to achieve the goal of stabilizing blood circulation and reducing the mortality of critically ill patients [10], such as CRRT reduces the mortality of patients with acute kidney injury and can effectively treat severe hyperkalemia [11, 12] and so on. CRRT has been increasingly applied to the treatment of HF, with many studies indicating its favorable efficacy in HF that is superior to conventional treatment; meanwhile, the application of nursing intervention has a positive effect on improving patient outcomes [13, 14]. However, little is known about the safety profile of this therapy in HT + RHF. Consequently, this paper evaluates the safety of CRRT in HT + RHF patients and analyzes the nursing highlights, to provide reliable evidence and methods for future clinical management of HT + RHF.

## 2. Materials and Methods

### 2.1. Study Area

The study was carried out of from March 2018 to February 2022.

### 2.2. Data Collection

With the approval of the Ethics Committee of our hospital, 66 HT + RHF patients admitted between March 2018 and December 2021 were enrolled and grouped as follows: a CRRT group with 33 cases treated with CRRT and a control group with 33 cases intervened by routine treatment. Additionally, all patients accepted individualized nursing strategies for blood purification tailored treatment formulated by our hospital. The eligible patients, all aged ≥50, met the diagnostic criteria of HT + RHF [15, 16] and agreed to receive CRRT treatment, with complete medical records, high compliance, and voluntary participation in this trial. In contrast, hospital referrals or those with communication barriers, physical impairment, other major diseases, infectious diseases, or short survival time were excluded.

### 2.3. Treatment Strategies

Control group: patients underwent a series of routine tests after admission. Their blood pressure (BP) and intracranial pressure were controlled to prevent complications. In addition to real-time monitoring of BP and blood oxygen, routine treatments such as cardiotonic, diuresis, vasodilator, and angiotensin-converting enzyme inhibitors were applied. Then, 25 mg sodium nitroprusside was added into 5% glucose solution for slow intravenous drip (6-12 drops/min), and the solution was changed every 6-8 hours. The treatment lasted for 14 days. CRRT group: based on the above treatment, patients in this group were given CRRT. The femoral vein double-lumen hemodialysis catheter was used to establish vascular access. All patients were treated with continuous veno-venous hemofiltration (CVVH), using AQU, Flex, ACH-10 pipelines, as well as MT-100, AEF-13, and HF1200 filters, with low molecular heparin anticoagulation as the main treatment. Each treatment lasted for 8 hours for a total of 14 days. Patients' vital signs, coagulation function, and electrolyte status were closely monitored, and corresponding adjustments were made according to patients' different reactions.

### 2.4. Nursing Strategies

Both groups received intensive care. After admission, the medical staff monitored the patients' BP, blood sugar, heart rate, and other vital signs three times a day and recorded them. In addition, health education was carried out for patients and their accompanying families to help them understand the disease, build up confidence, and improve treatment compliance. Furthermore, the medical staff paid attention to the presence of anxiety, nervousness, and other adverse emotions in patients and conducted timely communication and guidance to ease their mood and give them care and encouragement. Furthermore, the intravenous indwelling needle was selected when possible, the inspection of patients was strengthened, and the liquid medicine was replaced in time; oral care such as oxygen inhalation and sputum aspiration was provided for patients in need. Since infusion pump administration requires patients to stay in bed for a long time, HT + RHF patients have limited activities and are at high risk of pressure ulcers. Therefore, the nursing staff carried out a dynamic risk assessment of pressure ulcers and gave timely and reasonable interventions. What is more, the ward was ventilated regularly, and patients and their families were guided on standardized and reasonable diet, as well as infection prevention. Moreover, patients were encouraged to exercise moderately within their physical tolerance to prevent muscle atrophy. And according to the different needs of patients, corresponding intervention guidance was given in a timely manner until they were discharged from hospital.

### 2.5. Endpoints

The outcome measures were as follows [17]: (1) therapeutic effects (markedly effective: BP returned to normal, with alleviated HF symptoms and significantly improved cardiac function (CF); effective: the BP was significantly reduced, with certain improvement in HF symptoms and CF; ineffective: no obvious changes in BP, symptoms, etc., the total effective rate = (markedly effective + effective)/total × 100%); (2) alterations of CF indexes after treatment: left ventricular ejection fraction (LVEF), left atrial pressure (LAP), cardiac index (CI), stroke volume (SV); (3) serum levels of B-type natriuretic peptide (BNP), C-reactive protein (CRP), and mean arterial pressure (MAP) after treatment; (4) clinical indices: asthma relief time, heart rate recovery (HRR) time, edema resolution time, and hospitalization time; (5) incidence of ARs (incidence of ARs = number of adverse reactions/total number × 100%); (6) psychological quality and pain: psychological quality and pain before and after the intervention were assessed using the self-rating anxiety and depression scale (SAS and SDS) [18] and visual analogue scale (VAS) [19], respectively. The higher the SAS and SDS scores, the more severe the patient's anxiety and depression; the higher the VAS score, the more obvious the patient's pain.

### 2.6. Statistical Processing

Data processing employed SPSS22.0. The intergroup difference of count data (denoted by percentage) used the chi-square test. The quantitative data were given (mean ± standard deviation), and the *t* test and paired *t* test were used to analyze the data that conformed to a normal distribution. For all analyses, differences were significant when *P* values < 0.05.

## 3. Results

### 3.1. Summary of Results

CRRT group exhibited higher overall response rate and better CF than control group (*P* < 0.05), with lower BNP, CRP, and MAP levels, and shorter time of asthma relief, HRR, edema resolution, and hospitalization (*P* < 0.05); the incidence of ARs was similar (*P* > 0.05); for both groups, the scores of SAS, SDS, and VAS reduced statistically after treatment (*P* < 0.05).

### 3.2. Patients' General Information

Patients' general data, including age, BMI, course of HT, sex, exercise habits, living environment, and ethnicity, were collected. After statistical analysis, we found no statistical difference in general data between groups (*P* > 0.05, Table 1), confirming the experimental comparability of the two groups.

### 3.3. Therapeutic Effects of Two Groups

After treatment, the number of cases of markedly effective, effective, and ineffective in CRRT group was 18 (54.55%), 13 (39.39%), and 2 (6.06%), respectively, with an overall response rate of 93.94%, versus 75.76% in control group. Apparently, the therapeutic effect was statistically higher in CRRT compared with control group (*P* < 0.05, Table 2).

### 3.4. Alterations of CF Indexes after Treatment

After treatment, the LVEF of CRRT group was (36.84 ± 7.06)%, higher than that of (33.26 ± 7.49)% in control group (*P* < 0.05, Figure 1(a)); the LAP of CRRT and control group groups was (12.87 ± 4.69) mmHg and (17.54 ± 5.96) L/min/m^2^, respectively, indicating a significantly lower posttreatment LAP in CRRT group (*P* < 0.05, Figure 1(b)); the intergroup comparison of CI revealed a higher posttreatment CI in CRRT group compared with control group (*P* < 0.05, Figure 1(c)); finally, it can be seen that the SV value of CRRT group was (63.55 ± 9.70) mL, which was also higher when compared to control group (*P* < 0.05, Figure 1(d)).

### 3.5. Changes of Clinical Indices

The asthma relief time of CRRT and control groups was (3.7 ± 0.9) d and (5.9 ± 1.1) d, respectively, revealing notably faster asthma relief in patients treated with CRRT (*P* < 0.05, Figure 2(a)). The HRR time of CRRT group was (8.3 ± 1.2) d, shorter than that in control group (*P* < 0.05, Figure 2(b)). Comparing the edema resolution time, we also found that CRRT group took less time to resolve edema than control group (*P* < 0.05, Figure 2(c)). Shorter hospitalization time was also determined in CRRT group compared with control group (16.1 ± 2.4) d vs. (20.7 ± 1.8) d, with statistical significance (*P* < 0.05, Figure 2(d)).

### 3.6. Serum Indexes and MAP Levels in Both Groups after Treatment

The BNP levels in both cohorts were detected after treatment, and a notably higher BNP level was determined in CRRT group (529.00 ± 65.75) *μ*g/L compared with control group (*P* < 0.05, Figure 3(a)). Similarly, the CRP of CRRT group was (12.40 ± 1.33) mg/L, lower than that of the control group (*P* < 0.05, Figure 3(b)). Finally, the MAP were counted and the results determined a markedly lower MAP in CRRT group versus control group (*P* < 0.05, Figure 3(c)).

### 3.7. Incidence of ARs in Two Groups

According to statistics, no serious ARs occurred in both cohorts of patients during the treatment. In CRRT group, nausea and vomiting, abdominal pain, hypotension, and gingival bleeding were found in 1 case each, with a total AR rate of 12.12%; while in control group, the above ARs were observed in 2, 2, 0, and 1 case, respectively, with an overall AR rate of 15.15%. The two groups showed no statistical difference in the AR rate (*P* > 0.05, Table 3).

### 3.8. Alterations of Psychological Quality and Pain in Both Groups before and after Treatment

Both groups showed adverse emotions such as depression and anxiety and strong pain before treatment, with no evident difference in SAS, SDS, and VAS scores (*P* > 0.05). Nor were there any notable differences in the above scores between them after treatment (*P* > 0.05), but compared with the baseline (before treatment), the scores of SAS, SDS, and VAS in both groups reduced statistically (*P* < 0.05, Figures 4(a)–4(c)).

## 4. Discussion

CRRT, as a blood purification technology widely used in clinical practice, has achieved remarkable results in the cardiovascular field [20]. CRRT has been found to reduce cardiac load, stabilize CF, restore the body's (especially kidney) sensitivity to diuretics, and improve oxygen supply and RHF status [21]. Therefore, an in-depth exploration of the application of CRRT in RHF may provide a more reliable safety guarantee for RHF patients in the future.

In this study, we observed better therapeutic effects in RHF patients treated with CRRT, with significantly improved CF after treatment and shorter time of asthma relief, HRR, and hospitalization, confirming the excellent application effect of CRRT on RHF, which is consistent with the results of previous studies [22, 23]. Compared with routine hemodialysis treatment, CRRT can more effectively remove fluid and stabilize hemodynamics while regulating fluid balance through continuous and slow blood purification, with no obvious impact on the cardiovascular system [24]. Moreover, the hemofilters used in CRRT have the advantages of good compatibility, strong adsorption capacity, and permeability, allowing them to adsorb or remove inflammatory factors as well as small and medium molecular toxins, thus inhibiting the high decomposition state and keeping the balance of water, electrolyte, and acid-base [25]. At the same time, CRRT has the characteristics of favorable safety, high tolerance in patients, and high success rate of treatment and is simple to operate and can be implemented at the bedside, especially for critically ill patients [26]. It is pointed out that the long duration of routine hemodialysis has a great influence on hemodynamics and even the therapeutic effect and may cause arrhythmia, hypotension, and even aggravation of HF and other ARs [27]. This is also consistent with our findings, indicating that CRRT is more suitable for the treatment of RHF. Moreover, CRRT is shown to remove inflammatory mediators released in large quantities due to HF-induced cardiomyocyte injury and necrosis, protect the functions of cardiomyocytes and vascular endothelial cells, and promote the recovery of CF [28], which may be one of the reasons for the better improvement of patients with CRRT. Compared with previous research results [29, 30], the excellent therapeutic effect of CRRT can just make up for the limitations of insufficient clinical treatment plans and poor therapeutic effect for RHF at this stage and provide more reliable treatment services for RHF patients, guaranteeing life safety of RHF patients.

In addition, lower posttreatment BNP, CRP, and MAP were observed in CRRT group versus control group, which can also testify the improvement effect of CRRT on RHF. We believe that CRRT plays the role of solute clearance by means of convection and dispersion and introduces arteriovenous blood into the semipermeable membrane filter with good permeability, in which the small molecular weight solute and water can clear the solute and water through the pressure gradient on both sides of the semipermeable membrane, thus reducing the burden on heart and kidney, keeping blood in a balanced state, restoring myocardial elasticity, improving CF, and reducing the synthesis and release of BNP and inflammatory factors [31–34]. However, its specific mechanism needs to be confirmed by further studies. There was no difference in ARs between the two groups, which indicates that CRRT has good safety. However, an expanded sample size is also needed for confirmation. Finally, since the application of CRRT in RHF is not common at present, targeted nursing strategies are also the focus of clinical attention. Combined with previous research and nursing experience, this study mainly focused on the psychological state, pain, and rehabilitation training of patients treated with CRRT. The experimental results showed decreased scores of SAS, SDS, and VAS in both cohorts after treatment, which preliminarily indicated the successful implementation of the nursing program. Modern medical services are not only limited to the pathological treatment of patients' diseases but also need to pay attention to the physical and psychological rehabilitation of patients in an all-round way [35, 36]. Therefore, more meticulous, professional, and individualized nursing services play an extremely critical role in it [33, 37]. For RHF patients with more severe disease, difficult treatment and poor prognosis, it is more worthwhile to adopt a unique nursing strategy. The targeted care for CRRT in this study also successfully improved the patient's psychological state and reduced the patient's pain experience during treatment, which is of great significance to improving the current overall medical service. However, due to the lack of nursing guidelines for CRRT at present, there may still be room for improvement in this nursing program. Further research will be carried out on the nursing of RHF patients treated with CRRT.

In future studies, we also need to increase the number of cases and extend the study cycle to evaluate the impact of CRRT on patient outcomes and obtain more comprehensive results. At the same time, the improvement mechanism of CRRT on various functions of RHF patients is still worth further exploring, which will also be the focus of our follow-up research.

## 5. Conclusion

CRRT can effectively improve the therapeutic effect and CF of patients with HT complicated by RHF, with extremely high clinical application value.

## Figures and Tables

**Figure 1:** Alterations of CF indexes after treatment. (a) Comparison of LVEF between CRRT group and control group. (b) Comparison of LAP between CRRT group and control group. (c) Comparison of CI between CRRT group and control group. (d) Comparison of SV between CRRT group and control group. Note: ^#^ indicates that the difference between the two groups is statistically significant (*P* < 0.05).

**Figure 2:** Changes of clinical indices. (a) Comparison of asthma relief time. (b) Comparison of heart rate recovery time. (c) Comparison of edema resolution time. (d) Comparison of hospitalization time. Note: ^#^ indicates that the difference between the two groups is statistically significant (*P* < 0.05).

**Figure 3:** Serum indexes and MAP levels in both groups after treatment. (a) Comparison of BNP between CRRT group and control group. (b) Comparison of CRP between CRRT group and control group. (c) Comparison of MAP between CRRT group and control group. Note: ^#^ indicates that the difference between the two groups is statistically significant (*P* < 0.05).

**Figure 4:** Alterations of psychological quality and pain in both groups before and after treatment. (a) Comparison of SAS scores before and after treatment. (b) Comparison of SDS scores before and after treatment. (c) Comparison of VAS scores before and after treatment. Note: ^#^ indicates that there is a statistically significant difference between the same group and the same group before treatment (*P* < 0.05).

**Table 1:** General information.

	CRRT group (*n* = 33)	Control group (*n* = 33)	*χ* ^2^ or *t*/*P*
Age	69.5 ± 6.2	69.9 ± 6.0	0.266/0.791
BMI (KG/m^2^)	27.0 ± 2.5	27.8 ± 1.7	1.520/0.133
Duration of hypertension (years)	5.2 ± 2.0	5.4 ± 1.4	0.668/0.507
Gender			0.062/0.804
Male	19 (57.58%)	18 (54.55%)	
Female	14 (42.42%)	15 (45.45%)	
Exercise habits			0.061/0.806
Yes	17 (51.52%)	16 (48.48%)	
No	16 (48.48%)	17 (51.52%)	
Living environment			0.262/0.609
In the city	20 (60.61%)	22 (66.67%)	
In rural areas	13 (39.39%)	11 (33.33%)	
Nationality			0.569/0.451
Han nationality	30 (90.91%)	28 (84.85%)	
Minority	3 (9.09%)	5 (15.15%)	

**Table 2:** Clinical curative effects.

Group	*n*	Markedly effective	Effective	Ineffective	Overall response rate
CRRT group	33	18 (54.55%)	13 (39.39%)	2 (6.06%)	31 (93.94%)
Control group	33	10 (30.30%)	15 (45.45%)	8 (24.24%)	25 (75.76%)
*χ* ^2^					4.243
*P*					0.039^a^

**Table 3:** Adverse reactions of two groups.

Group	*n*	Feel sick and vomit	Stomach ache	Low blood pressure	Bleeding gums	ARs
CRRT group	33	1 (3.03%)	1 (3.03%)	1 (3.03%)	1 (3.03%)	4 (12.12%)
Control group	33	2 (6.06%)	2 (6.06%)	0 (0.00%)	1 (3.03%)	5 (15.15%)
*χ* ^2^						0.129
*P*						0.720

## Data Availability

The data presented in this study are available upon request from the corresponding author.
